# Establishing a Regulatory Science System for Supervising the Application of Artificial Intelligence for Traditional Chinese Medicine: A Methodological Framework

**DOI:** 10.1155/2022/9680203

**Published:** 2022-06-02

**Authors:** Ying He, Qian Wen, Ying Wang, Juan Li, Ning Li, Rongjiang Jin, Nian Li, Yonggang Zhang

**Affiliations:** ^1^Department of Integrated Traditional and Western Medicine, West China Hospital, Sichuan University, Chengdu, China; ^2^Department of Medical Administration, West China Hospital, Sichuan University, Chengdu, China; ^3^School of Health Preservation and Rehabilitation, Traditional Chinese Medicine of Chengdu University, Chengdu, Sichuan, China; ^4^Department of Periodical Press, West China Hospital, Sichuan University, Chengdu, Sichuan, China; ^5^Department of Evidence-based Medicine and Clinical Epidemiology, West China Hospital, Sichuan University, Chengdu, China

## Abstract

In this study, we reported a methodological framework for the development of a guideline for establishing a regulatory science system for supervising the application of artificial intelligence for traditional Chinese medicine (TCM). It introduced all of the key steps for developing the guideline as follows: the composition of the guideline expert groups, summary steps, agency, purpose, targeted population, writing, publishing, updating, dissemination, dynamic monitoring, and evaluation. The guideline will provide the basis for national authorities to effectively regulate artificial intelligence technology and enrich the supervisory system for TCM, and it will be of great significance to TCM.

## 1. Introduction

Traditional Chinese medicine (TCM) is a medical and pharmaceutical system with a long history, unique theory, and technical methods, which made great contributions to human health [1]. As a result of dissemination of TCM, domestic and foreign scholars have conducted many scientific research studies, and its influence has gradually expanded [2, 3]. Many landmark research studies have been published in top journals, including Journal of the American Medical Association (JAMA), Annals of Internal Medicine, and JAMA Internal Medicine [4–6]. Thus, the academic influence of TCM has greatly improved. However, its international influence is still encountering challenges, which are mainly reflected in the reluctance of some disciplines to accept the validity of the recognition of TCM [7, 8].

As a result of the development of computer science, the application of artificial intelligence (AI) can effectively transform the combined online and offline medical model to achieve multidisciplinary integration, multipath diagnosis, and treatment of the wisdom of the Internet medical, which can improve the efficiency of diagnosis, treatment, and management [9, 10]. In recent years, interest in AI has increased in the application of data mining, computer-aided diagnosis, intelligent decision therapy, and intelligent rehabilitation of TCM [11]. AI can convert TCM's classical ancient books and clinical treatment experience into data and establish an extremely large TCM database to provide a basis for scientifically explaining TCM treatments. Doing this can greatly improve the overall service level of TCM, reduce the number of medical resources required, and promote the development of TCM [12, 13].

As a result of the wide application of AI technology in the construction of an evaluation system, disease model construction, medical device innovation, and public health crisis response, the establishment of a regulatory science system for supervising the application of AI has become a potential research topic [14, 15]. Until now, no such study has been conducted in this field, and no such guideline has been developed, and it is urgent to develop a guideline in this field. Thus, we will develop such a guideline. In order to make the guideline transparent [16, 17], we reported the current methodological framework. It will help to establish a regulatory science system and to help in the application of AI technology to TCM. It will also fill research gaps and help TCM serve human health [18].

## 2. Methods

### 2.1. Summary Steps of Developing Guideline

The guideline's development will follow the latest definitions of guidelines provided by the United States Institute of Medicine [19], which are based on the methodology developed by the World Health Organization standard guidance [20] and the six major areas of the Appraisal of Guidelines for Research and Evaluation (AGREE II) [21]. We will also use the Reporting Items for Practice Guidelines in Healthcare (RIGHT) [22] and other international standards to help us develop the guideline [23–26]. The key steps of the guideline are shown in Figure 1.

The development of the guideline consists of four phases (Figure 1). In phase 1, we will form the guideline groups and construct the problems and outcomes. Additionally, we will survey experts from universities and scientific research institutions. In phase 2, we will conduct a systematic review of all available guidelines, documents, and papers on supervising the application of AI to TCM and provide evidence for developing items of the guideline. In phase 3, first, we will draft the initial version of the guideline based on the results from the Delphi method and consensus meeting. Subsequently, we will modify, validate, and finalize the guideline through multiple steps. In phase 4, we will establish the regulatory scientific evidence base, dynamic update, and evaluation protocol.

### 2.2. Explanations of the Terms

TCM [27]: traditional Chinese medicine (TCM) is an alternative medical practice drawn from traditional medicine in China. It includes various forms of herbal medicine, acupuncture, cupping therapy, Guasha, massage (Tuina), bonesetter (Die-Da), exercise (Qigong), and dietary therapy.

AI [28]: artificial intelligence (AI) is a broad umbrella term used to encompass a wide variety of subfields dedicated to creating algorithms to perform tasks that mimic human intelligence. It combines human abilities of learning, reasoning, perception, and an understanding of natural language through computer programs.

Regulatory science [29]: regulatory science is the science of developing new tools, standards, and approaches derived from various scientific disciplines to assess the safety, efficacy, quality, and performance of all Food and Drug Administration (FDA)-regulated products.

Living guideline [30]: A living guideline is a novel approach that operates through, for example, dynamic monitoring, timely inclusion of new evidence, and live updates of recommendations to effectively improve the timeliness of clinical guidelines by periodically obtaining clinical evidence and updating the results of systematic reviews in a timely manner.

### 2.3. Ethics and Dissemination

The guideline will not require ethical approval because no data linked to individual patient information will be used in our study. Additionally, the findings will be disseminated through peer-reviewed journals or conferences.

### 2.4. Agency of the Guideline

The guideline will be developed by members from editorial boards of the Journal of Evidence-Based Medicine and the Chinese Journal of Evidence-Based Medicine, in collaboration with a large number of institutions in China, and we will invite experts from multiple units outside of China.

### 2.5. Guideline Teams

The guideline teams consist of a guideline steering committee, guideline expert group, guideline secretariat group, and external review group. To ensure the authority and comprehensiveness of the guideline, the guideline teams will include experts from main cities around China. Additionally, we will invite regulatory science experts from countries out of China to participate. Members of the guideline steering committee, guideline expert group, guideline external review group, and secretariat group should complete a declaration of interest and declare any conflict of interests before formally participating in the work related to the development of the guideline. All members' statements of interest will be reported in the final guideline document.

### 2.6. Patient and Public Involvement Statement

The current study is a methodological study, and patient and public involvement is not needed.

### 2.7. Purpose and Targeted Population of the Guideline

The purpose of the guideline is to establish a regulatory science system for supervising the application of AI to TCM. The guideline will focus on the scientific regulatory approach, comprehensive evaluation, and dynamic updating of the application of AI to TCM. This guideline applies to personnel at all levels who conduct regulatory science research on the application of AI to TCM, including policy-makers, medical device managers, clinicians, nurses, computer scientists, and journal editors.

### 2.8. Clarify the Guideline Questions

Guiding questions will be designed by the guideline steering committee using the relevant literature and study objectives. A three-round Delphi study will be conducted to determine the issues that refer to the guidance and the development method of the regulatory scientific system. Each item will be rated by using a five-point Likert scale (not important, of little importance, neutral, important, and very important). The mean value (*X*), standard deviation (SD), coefficient of variation (CV), and *R* value will be calculated for each attribute.

### 2.9. Search Strategy

The search databases will include PubMed, the Cochrane Library, Embase, Chinese Biomedical Literature Service System, China National Knowledge Infrastructure, WanFang Data, China Science and Technology Journal Database, UptoDate, Guideline Central, National Guideline Clearinghouse, Guidelines International Network, and the National Institute for Health and Care Excellence. The following databases will also be searched: NHS Economic Evaluation Database and Health Technology Assessment. Additionally, information will be obtained from official websites, such as the health authorities' official websites of the international and local organizations anduniversities, Food and Drug Administration, and the official website of the health insurance department or relevant industry association. Finally, we will search Google, Baidu, and other search engines to obtain other literature. According to the retrieval strategy formulated in advance, articles from the above databases will be imported into the Endnote X9 software.

Subject words and text words will be searched. Search terms will include guideline, consensus, standard, process, artificial intelligence, machine learning, traditional Chinese medicine, TCM, regulatory science, and handbook. There will be no limitation to the types of included studies. The languages will be limited to English and Chinese. The search will be performed in May 2022, and the search will be updated when necessary.

### 2.10. Survey of Problems

We will conduct a survey of problems from TCM universities and research institutions regarding the application of AI to TCM. It will help us to understand the current scenario and problems regarding the application of AI to TCM.

### 2.11. Literature Screening and Data Extraction

To achieve the stability and consistency of literature retrieval, preretrieval will be performed to achieve a unified standard. The inclusion criteria will be as follows: any study that is helpful to establish a regulatory science system for the application of artificial intelligence in TCM, including guideline, consensus, standard, process, article, or review. The exclusion criteria will be as follows: the study does not report the clear method for establishing a guideline; it does not involve a regulatory science system. When necessary, the criteria will be revised. Two researchers will independently select and screen the studies according to inclusion criteria and exclusion criteria. A third researcher will be consulted to resolve the disagreement. These two researchers will independently extract data, and discrepancies will be resolved by consensus. If information cannot be retrieved, the corresponding author will be contacted.

### 2.12. Systematic Review

The quality of the included studies will be assessed according to the types of studies. The risk of bias (ROB) will be assessed using ROB 2.0 for RCTs [31]. The Newcastle–Ottawa Scale [32] will be used to assess the quality of cohort studies or case-control studies. The AGREE II will be used to assess the quality of guidelines [33]. A Measurement Tool to Assess Systematic Reviews 2 (AMSTAR 2) will be used to assess the quality of systematic reviews and meta-analyses [34]. The process will be performed by two independent researchers. Disagreement will be discussed or consulted by a third researcher. A systematic review will be performed to assess the potential studies and to provide evidence to develop the guideline. It will also help to provide recommendations for the guideline.

### 2.13. Generation of a List of Candidate Items

The candidate items in the guideline will be developed using the Delphi method. We will develop the candidate items before sending them the questionnaire. A two-round Delphi questionnaire and a final consensus meeting will be employed [35, 36]. An item will be recommended if the votes are above 50%. The remaining scenarios will be considered if no consensus is reached, and recommendations with no consensus will be subjected to the next round of voting. A subsequent review of the results will be conducted by the steering committee to identify statements where a consensus is almost reached. With the agreement of two-thirds of the members of the consensus expert group, the steering committee may revise and improve important issues existing in the recommendations, and the guideline secretariat group will faithfully record the entire revision process.

### 2.14. Writing, Publishing, and Updating the Guideline

Once the recommendations are approved, the guideline steering committee will write the guideline according to the RIGHT (http://right-statement.org) reporting standard. The draft guideline will be submitted to the steering committee for review and approval. Then, the introduction and announcement of the guideline will be published. The guideline will also be presented and discussed at relevant professional society academic meetings and through publication in scientific journals. We will establish the regulatory scientific evidence systematic based on the guideline. The guideline will be updated according to the feedback on the actual operation of the guideline and the latest research results in relevant fields.

## 3. Discussion

Developing a guideline for establishing a regulatory science system for supervising the application of AI to TCM is urgent because the development of AI is so fast. The future guideline will be developed by a multidisciplinary team of experts. To help the guideline, opinions will be obtained from experts, policy-makers, and users. The guideline developers will establish an update and evaluation process to update the guideline and finally help supervise the application of AI in TCM. The guideline will not only track new evidence in real time, promote the practical application of the best research evidence, and implement scientific regulation but also save a large number of resources and optimize the guideline formulation and evaluation process. The guideline will be a new innovation in TCM.

In conclusion, the current study describes the steps of formulating a guideline for the application of AI to TCM. The guideline will be developed in strictly accordance with the standards of an evidence-based guideline. The results will be used as a context for analyzing general strengths and gaps in the current quality of evidence in the application of AI to TCM.

## Figures and Tables

**Figure 1:** Key steps of methodology of the guideline.

## Data Availability

The data used to support this study are included within the article and available from the corresponding author upon request.
